The article "Human-Computer Interaction with Hand Gesture Recognition Using ResNet and MobileNet" was published in 2022. Journal: Comput Intell Neurosci.

# Human-Computer Interaction with Hand Gesture Recognition Using ResNet and MobileNet

**DOI:** 10.1155/2022/8777355

**Published:** 2022-03-26

**Authors:** Abeer Alnuaim, Mohammed Zakariah, Wesam Atef Hatamleh, Hussam Tarazi, Vikas Tripathi, Enoch Tetteh Amoatey

**Affiliations:** ^1^Department of Computer Science and Engineering, College of Applied Studies and Community Services King Saud University, P.O. Box 22459, Riyadh 11495, Saudi Arabia; ^2^Department of Computer Science, College of Computer and Information Sciences, King Saud University, P.O. Box 51178, Riyadh 11543, Saudi Arabia; ^3^Department of Computer Science and Informatics, School of Engineering and Computer Science, Oakland University, 318 Meadow Brook Rd, Rochester, MI 48309, USA; ^4^Department of Computer Science & Engineering, College of Graphic Era Deemed to be University, Dehradun, Uttarakhand, India; ^5^School of Engineering, University for Development Studies, Tamale, Ghana

## Abstract

Sign language is the native language of deaf people, which they use in their daily life, and it facilitates the communication process between deaf people. The problem faced by deaf people is targeted using sign language technique. Sign language refers to the use of the arms and hands to communicate, particularly among those who are deaf. This varies depending on the person and the location from which they come. As a result, there is no standardization about the sign language to be used; for example, American, British, Chinese, and Arab sign languages are all distinct. Here, in this study we trained a model, which will be able to classify the Arabic sign language, which consists of 32 Arabic alphabet sign classes. In images, sign language is detected through the pose of the hand. In this study, we proposed a framework, which consists of two CNN models, and each of them is individually trained on the training set. The final predictions of the two models were ensembled to achieve higher results. The dataset used in this study is released in 2019 and is called as ArSL2018. It is launched at the Prince Mohammad Bin Fahd University, Al Khobar, Saudi Arabia. The main contribution in this study is resizing the images to 64 ∗ 64 pixels, converting from grayscale images to three-channel images, and then applying the median filter to the images, which acts as lowpass filtering in order to smooth the images and reduce noise and to make the model more robust to avoid overfitting. Then, the preprocessed image is fed into two different models, which are ResNet50 and MobileNetV2. ResNet50 and MobileNetV2 architectures were implemented together. The results we achieved on the test set for the whole data are with an accuracy of about 97% after applying many preprocessing techniques and different hyperparameters for each model, and also different data augmentation techniques.

The article "Human-Computer Interaction with Hand Gesture Recognition Using ResNet and MobileNet" was published in 2022. Journal: Comput Intell Neurosci.

## 1. Introduction

Human-computer interaction (HCI) has now become a frequent element of our lifestyles as computer technology and hardware equipment have advanced. The usage of hand signals in this HCI has piqued people's curiosity since it is a nice method of engaging with the computer [1, 2]. A hand gesture is a means of expressing yourself via the motion of your palm and fingers [3]. Hand gesture can be used to interface with devices in HCI, eliminating any need for the additional input device. A person's gesture must be recognized by a device for effective dialogue between a human and a computer. As a result, HGR has grown in importance as a study issue and a requirement in today's environment [4], robot control [5], virtual gaming [6], and natural user interfaces is just a few of the applications [7]. A well-known use of hand gesture recognition is the identification of human data, namely, sign language [8, 9]. Sign language is a visual language in which ideas are communicated by a series of expressive hand motions in a certain order [10]. For deaf people, it is their only means of communication. According to the World Health Organization (WHO), 5% of the world's population (about 360 million people) has moderate to severe hearing loss and can only communicate via their local sign language (WHO, 2015). Because this communication is difficult for the auditory population to grasp, there is a communication gap between the normal and speech-hearing impaired groups. As a result, computer-assisted gesture detection may be used to translate between sign languages. This would be beneficial and would act as a bridge between the two communities. Fixed movements and dynamic gestures are the two forms of sign language hand motions. Static gestures are described as the placing of hands and fingers in a fixed position with no movement in relation to time, whereas dynamic gestures are defined as hands moving in a continuous motion in relation to time. There are two methods for identifying hand gestures for sign language translation: vision-based and glove-based [11, 12]. Some of the latest works are on hand gesture recognition, which are recently published [9, 13, 14]. Electronic equipment such as data collection, accelerometers, bands, and other similar devices must be worn by participants in the contact-based method. These components detect changes in motion and transmit the data to a computer for further analysis. Although this strategy has received positive feedback in the research [15], it is costly and time-consuming for ordinary human-computer interaction interface operators. Because the signer's data are recorded using a camcorder, the vision-based technique may be more user-friendly. By analyzing data acquired through image processing algorithms, this technology decreases users' reliance on sensory equipment. This study discusses a vision-based technique for recognizing static hand movements for a sign language translation system. A novel and reliable method based on convolutional neural networks (CNNs) has been developed for this purpose. VGG-11 and VGG-16 have been improved and deployed for gesture recognition in addition to the suggested technique.

The article "Human-Computer Interaction with Hand Gesture Recognition Using ResNet and MobileNet" was published in 2022. Journal: Comput Intell Neurosci.

The list of contributions in this study is as follows:

- The images are resized to 64 ∗ 64 pixels and converted from grayscale images to three-channel images.
- We applied the median filter to the images, which acts as lowpass filtering in order to smooth the images and reduce noise.
- To make the model more robust when generalizing in real-life scenarios (images) and also to avoid overfitting as possible, different augmentation techniques are applied to the images.
- Then, the preprocessed image is fed into two different models, which are ResNet50 and MobileNetV2.
- ResNet50 and MobileNetV2 architectures were implemented together.

The remaining of the study is organized as follows: Section 2 gives the literature addressing the problem and the technique applied to solve the sign language recognition issue, and then, Section 3 gives the details of the dataset and different preprocessing techniques.  Section 4 describes the methodology applied with proper architecture design, and Section 5 gives the results with comparative analysis followed by Section 6 with conclusions followed by the list of references.

## 2. Literature Review

For sign language recognition in the human-computer relationship, many approaches are present in the literature. The basic goal of these technologies is to facilitate communication by deducing the accurate interpretation of the user's gestures/signs. The following steps are included in this methodology: capture and preprocessing, gesture representation, feature extraction, and categorization. This subject looks at various movement recognition techniques in the framework of several sign languages. A summary of these strategies is provided below.

ASL Akhter (2018) described a technique for recognizing ASL alphabets. The multiple ASL alphabets are represented using PCA-based attributes, a Gabor filter, and orientation-based hash values. The collected characteristics are then categorized to use an artificial neural network (ANN). The effectiveness of their self-created database of 24 fixed motions was examined in this study. Similarly, the authors in this study [16] have created a CNN-based model for human gesture recognition. For this, the model is trained and evaluated on 31 distinct ASL alphabet and number classes. In another work [17], the authors have used a different approach of ASL alphabet identification in which both color and depth pictures of gestures were supplied into a CNN model. In this model, two convolutional layers are utilized to extract characteristics from every intake, and the information from these levels is combined and sent for categorization into a fully connected layer. In addition to RGB photographs, numerous academics have worked using depth sensors such as the Microsoft Kinect. In this study [18], the authors have demonstrated a technique for sign language recognition utilizing CNN with multiview augmentation and reasoning fusion. The depth photographs of the motions were collected using the Microsoft Kinect camera. The writers of this study proposed using augmented data for CNN model coaching. This approach obtained high classification accuracy at the expense of high computation complexity. Additional Kinect sensor-based hand gesture recognition method for ISL identification has been seen in the research [19]. In this study, a research was conducted by employing a distinct mix of feature extraction and machine learning techniques for accurate recognition of hand gestures. A total of 140 static words were used to measure performance across a variety of classes. In another work [20], the authors described a new approach for recognizing ASL fingerspelling that makes use of a depth sensor. The writers used a principal component analysis network (PCANet) to retrieve and learn features from depth images in this document. Lastly, a linear SVM (support-vector machine) is used to classify 24 static ASL motions. Authors here [21] have suggested a method for recognizing ISL using a 5-layer CNN model. The information in this study was collected from 12 distinct signers that use the Microsoft Kinect sensor. This method's performance has only been evaluated for ISL numerals and alphabets.

The article "Human-Computer Interaction with Hand Gesture Recognition Using ResNet and MobileNet" was published in 2022. Journal: Comput Intell Neurosci.

For gesture recognition, several writers in journals have employed contact-based approaches. Authors here [22] have presented a wearable gadget-based approach for detecting ASL. Six inertial measuring units (IMUs) were used to create 28 ASL sentences, which were then classified using the LSTM algorithm. For a Chinese sign language translation system, Xiao et al. propose a movement detection strategy based on recurrent neural networks (RNNs). The signer's skeleton pattern is employed for bidirectional communication in this investigation. The performance of this approach is assessed using standard RGB depth images of various stationary movements. For ISL translation, [23] demonstrated a sensor-based real-time hand gesture detection system.

For segmentation, Zernike moments and SVM were utilized. Reference [24] showed a solution for static gesture recognition using Inception V3. For performance evaluation, the static image dataset of 24 English letter ASL from [25] was used. Using Inception v3, a 2-stage learning approach was used to fine tune the classification model, which achieved an efficiency of 91.35 percent. A neural network-based SLR approach was described by the researchers of [26]. A hand-detecting network based on faster R-CNN and 3D CNN for extracting features, and LSTM for encoding and decoding make up the whole identification system. Despite the fact that the dataset is limited, this method yields good identification accuracy. For SLR systems, [27] proposed a deep learning-based architecture. A CNN-based framework was used for the classification of the indications. A web camera-based database of ISL alphabets, numerals, and phrases was used to assess performance in this study. The productivity of this technique was examined using different optimizers in the CNN architecture. Contact-based, Kinect-based, and RB image-based hand motion recognitions are all evaluated in Table 1. The following conclusions may be taken from this section's literature review.

The authors in this study [28] have proposed an Arabic sign language recognition and generating Arabic speech system, they worked on a dataset, which they manually collected, the dataset has 31 classes 125 pictures for each 31 alphabet classes, and the suggested system is diﬀerently tested by combining hyperparameters to obtain the optimal outcomes with the least training time. They applied different preprocessing techniques such as the extracted images are resized to 128 × 128 pixels and converted to RGB and applied different augmentation techniques such as rotating images, horizontal flipping, and shearing images with 0.2 random degree range. They used a CNN model for feature extraction and classification, and the model was trained on 80% of the dataset and tested on 20% rest of the dataset and achieved 90% accuracy on the test set.

Sagayam and Hemanth [4] proposed an Arabic sign language recognition made by a group of researchers from the Umm Al Qura University, Saudi Arabia, they worked on ArSL (2018) dataset, they applied some preprocessing techniques such as removing noise from image, converting images to gray scale, resizing them to dimensions 64 ∗ 64 pixels and normalizing them by dividing each pixel on 255 to convert the range of pixels from 0 to 255 to 0–1, they proposed a custom CNN model, which was trained on 80% of the data and tested on the remaining 20% (11,089 images), the accuracy they achieved on the training set was 98.06%, and the accuracy they achieved on the test set was 88.87%.

The article "Human-Computer Interaction with Hand Gesture Recognition Using ResNet and MobileNet" was published in 2022. Journal: Comput Intell Neurosci.

In [29], as an example, a team of academics from the Al-Azhar University in Cairo, Egypt, and the King Khalid University in Abha, Saudi Arabia, presented an Arabic sign language recognition system for alphabets using machine learning methods. They experimented on a collection of 2,800 photographs and 28 classes, with 10 persons considering the 28 distinct alphabets. Each letter received 100 photographs, for a total of 2,800 pictures. Color photographs are enhanced in order to increase picture value. The color picture is transformed to grayscale picture with 256 density stages and then resized to 640 x 480 pixels. Filtering techniques are also used to reduce ambient sound. They additionally conducted optimization and picture improvement algorithms, classification, and morphological straining to the color photograph in a variety of methods to produce the best example to enable us subsequently retrieve one of the best attributes and achieve the greatest efficiency. The feature extraction is performed using hand shape-based description, where each hand image was described by a vector consisting of 15 values where the values represent the key point locations, and the classification part was performed by some algorithms such as, KNN classifier, Naïve-Bayesian, and MLP. When testing, they achieved an accuracy rate of 97.548%.

## 3. Dataset

The dataset used is called ArSL2018 [30] launched at the Prince Mohammad Bin Fahd University, Al Khobar, Saudi Arabia, to be made available to machine learning and deep learning researchers. The dataset consists of 54,049 images for the 32 Arabic sign language sign and alphabets (32 classes), and Figure 1 shows a sample of each Arabic sign language alphabet in this dataset. Each class is named in English, and each class images vary from about 1,300 to 2,200 images, and Table 1 shows the classification of the Arabic alphabet signs, with labels and number of images.

In Figure 2 below, we can see the distribution of the classes in our dataset.

### 3.1. Dataset Limitations

1. The whole dataset was captured in a single location and on a similar background.
2. There are not enough orientations, and most images in each class are taken in the same pose.
3. Not enough noise, lightning, and zooming variations were introduced in the classes of the dataset.
4. The number of contributors providing the sample images was limited.
5. The number of images differs from one class to another (imbalanced classes) as shown in Figure 2.

The article "Human-Computer Interaction with Hand Gesture Recognition Using ResNet and MobileNet" was published in 2022. Journal: Comput Intell Neurosci.

### 3.2. Data Preparation and Preprocessing

Data preprocessing is the first step before building a deep learning model. It is used to transform the raw data in a useful and efficient format.

#### 3.2.1. Formatting Images

The images are resized to 64 ∗ 64 pixels and are converted from grayscale images to three-channel images, which are observed by stacking three grayscale channels to form the image, in order to be compatible with applying transfer learning with some models.

#### 3.2.2. Noise Removal and Image Smoothing

We applied the median filter to the images, which acts as lowpass filtering in order to smooth the images and reduce noise. The median filter is effective at removing noise while preserving edges and features of the image.

### 3.3. Data Augmentation

The dataset images have many limitations as we discussed briefly in the dataset section, since all the images of the dataset nearly fall on the same distribution due to the lack of variety in the images, so we used different augmentation techniques in order to somehow address this problem, to make the model more robust when generalizing in real-life scenarios (images) and also to avoid overfitting as possible. Different augmentation techniques are applied to the images such as horizontal flip, different rotation angles, shearing, and different brightness ranges shown in Figures 3–6 respectively, random rotations are applied on images from 0 to 30° to address the problem of fixed orientations as possible, and random brightness ranges were applied in order to make the model invariant to different illuminations. The function used to do these operations is image flips via the horizontal_flip and vertical_flip arguments, and rotation_range argument brightness_range argument.

### 3.4. Splitting Dataset for Training and Testing

A ratio of 80 :  20 is used for dividing the dataset into training and testing set, where the constructed models were trained on around 44,000 images and tested on around 10,000 images.

## 4. Methodology

First, the hand is detected from the frames of the video using OpenCV, then the detected region of interest that surrounds the hand is cropped from the frame, then we apply our preprocessing techniques to the cropped hand, then the obtained cropped image is converted from RGB to gray scale, then the image is resized into dimensions 64 ∗ 64, then our obtained gray-scale image is converted into a three-channel image by stacking the gray-scale channel 3 times to obtain our 64 ∗ 64 ∗ 3 image as we trained our models on these dimensions, then we apply the median filter to our image to reduce noise and smooth the image, and then, the preprocessed image is fed into two different models, which are ResNet50 and MobileNetV2.

The article "Human-Computer Interaction with Hand Gesture Recognition Using ResNet and MobileNet" was published in 2022. Journal: Comput Intell Neurosci.

### 4.1. ResNet50 Architecture

ResNet, short for residual networks, is a traditional neural network that helps as the basis for several computer vision applications. The essential invention with ResNet was that it empowered us to successfully train extraordinarily neural networks. Prior to ResNet, very deep neural networks were hard to train due to the issue of vanishing gradient problem.

Therefore, just tallying layers together does not work to upsurge system complexity. Deep networks are tough to train because of the well-known disappearing gradient problem. When the gradient is backpropagated to older levels, repetitive multiplication can lead the gradient to become incredibly tiny. When a consequence occurs, as the network deeply penetrates, its functionality becomes overwhelmed or even begins to degrade fast.

When we get deeper into the model a problem occurs called vanishing gradient. So, ResNet helps in countering this issue which is its main strength. ResNet accomplishes this by applying skip connection technique. So, ResNet main strength is skip connection.

ResNet was the first to establish the notion of a skip connection. The skip link is seen in the two pictures beneath. The picture on the left, Figure 7, shows convolution layers being sequentially loaded. On the right, Figure 8, we endure to build obscurity layers as previously, but we now embrace the original data to the convolution block's output.

This identity mapping (skip connection) between layers adds the outputs from previous layers to the output of the layers ahead. This results in the ability to train much deeper networks than what was previously possible. The detailed building block of ResNet is shown in Figure 9.

Our modified ResNet50 architecture layers, hyperparameters, optimizer, etc. are shown in Table 2.

### 4.2. MobileNetV2 Architecture

Based on an architecture that uses depthwise separable convolutions to build lightweight deep neural networks, computation, and size trade-offs of shrinking the MobileNetV2 architecture with the width multiplier, Figure 10 shows the building block of MobileNetV2.

We all know that there are some operations that have a higher cost than other operations, for example, multiplication operation has a much higher cost than addition. Standard convolution is very costly as all its operation is multiplication as shown in Figure 11. Suppose there are N filters/kernels of size Dk × Dk × M. If a normal convolution operation is done, then the output size will be as shown in Equation (1). So, for normal convolution operation, total no of multiplications will be as shown in Equation (2). A single convolution operation requires Dk × Dk multiplications. Then, the total number of multiplications is equal to as shown in Equation (3). So,

(1) $$\begin{array}{c} \text{Total no of multiplications}=M\times D_{k}^{2}\times D_{p}^{2}D_{p}\times D_{p}\times N, \end{array}$$

(2) $$\begin{array}{c} N\times D_{p}^{2}\times D_{k}^{2}\times M, \end{array}$$

(3) $$\begin{array}{c} M\times D_{p}\times D_{p}\times D_{k}\times D_{k}. \end{array}$$

(4) $$\begin{array}{c} \text{Mult sonce}=D_{K}^{2}\times M, \end{array}$$

(5) $$\begin{array}{c} \text{MultsperKernel}=D_{G}^{2}\times D_{k}^{2}\times M, \end{array}$$

(6) $$\begin{array}{c} \text{MultsNKernels}=N\times D_{G}^{2}\times D_{k}^{2}\times M. \end{array}$$

So MobileNet reduces the multiplication operation that happens in normal convolution, as MobileNet follows two main stages, which are depthwise convolution stage shown in Figure 12 and pointwise convolution stage shown in Figure 13 instead of standard convolution.

The article "Human-Computer Interaction with Hand Gesture Recognition Using ResNet and MobileNet" was published in 2022. Journal: Comput Intell Neurosci.

Depthwise convolution:

Pointwise convolution:

In the equations below, the detailed operations are discussed, which is used by MobileNet during the convolution stages. It is supposed there are input data of size *D*_*f*_ × *D*_*f*_ × *M*, where *D*_*f*_ × *D*_*f*_ can be the image size and *M* is the number of channels (3 for an RGB image). It is supposed that there are *N* filters/kernels of size *D*_*k*_ × *D*_*k*_ × *M*. If a normal convolution operation is performed, then, the output size will be *D*_*p*_ × *D*_*p*_ × *N* as shown in equations (7)–(9).

In depthwise convolution step (the first step in filtering stage):

(7) $$\begin{array}{c} \text{Multsonce}=D_{k}^{2}, \end{array}$$

(8) $$\begin{array}{c} \text{Mults}1\text{channel}=D_{G}^{2}\times D_{K}^{2}, \end{array}$$

(9) $$\begin{array}{c} \text{DCMults}=M\times D_{G}^{2}\times D_{K}^{2}, \end{array}$$

In pointwise convolution step (the second step in filtering stage):

In pointwise operation, a 1 × 1 convolution operation is applied on the M channels. So, the filter size for this operation will be 1 × 1 × *M*. To say, we use *N* such filters, the output size becomes *D*_*p*_ × *D*_*p*_ × *N,* as shown in equations (10)–(13) that give the total value.

(10) $$\begin{array}{c} \text{Multsonce}=M, \end{array}$$

(11) $$\begin{array}{c} \text{Mults}1\text{channel}=D_{G}\times D_{G}\times M\text{,} \end{array}$$

(12) $$\begin{array}{c} \text{PCMults}=N\times D_{G}\times D_{G}\times M\text{,} \end{array}$$

(13) $$\begin{array}{c} \text{Total}=\text{DCMults}+\text{PCMults.} \end{array}$$

Our modified MobileNetV2 architecture layers, hyperparameters, optimizer, etc. are shown in Table 3.

The article "Human-Computer Interaction with Hand Gesture Recognition Using ResNet and MobileNet" was published in 2022. Journal: Comput Intell Neurosci.

### 4.3. Our Whole Proposed Methodology

1. The person hand is detected in each frame of the camera video in real time and the region of interest, in which the human hand is cropped from the video frame.
2. Our preprocessing techniques are applied to our cropped hand image, which are as follows: resizing the image into 64 ∗ 64, converting the image to gray scale, applying a median filter with size 3 ∗ 3 for removing the salt and pepper noise generated by the camera and for image smoothing, and stacking 3 of the grayscale image to form an image of dimensions 64 ∗ 64 ∗ 3 to be compatible with what the model was trained on.
3. After the hand image is cropped and preprocessed, it is fed to two models, which are as follows: ResNet50 and MobileNetV2 are pretrained on the ImageNet dataset in order to take the advantage of transfer learning instead of beginning the model weights with random initializations. The features extracted from each model (ResNet50 and MobileNetV2) are flattened into a 1D feature vector and then entered into the fully connected layers, which is responsible for the classification part, the first layer of the fully connected layers consists of 1,024 neurons, the second layer consists of 512 neurons, and then, our last layer is the softmax layer, which distributes probabilities among the 32 Arabic sign language alphabet classes. The hyperparameters, architecture, optimizers, etc. of the two models (ResNet50 and MobileNetV2) are discussed above in detail in Tables 2 and 3, respectively.
4. Each of the two models used will return its predictions. Those predictions are ensembled by averaging the predictions of the two models. At the end, the alphabet class with the maximum average prediction is returned as the classified alphabet class.

The whole methodology we talked about is briefly shown in Figure 14.

## 5. Results

The performance of the hand sign recognition system is evaluated using the test set where the dataset is split, which consists of 54,000 images with a ratio of 80% training set to 20% test set, which is around 44,000 samples to 10,000 samples, and our results are based on these 10,000 sample.

The two models (ResNet50 and MobileNetV2) we used achieved accuracies that range from 96% to 98%, and Figure 15 shows the accuracy of the training vs the accuracy of the validation among 10 epochs on the ResNet50 model, while in Figure 16 shows the loss of the training vs the loss of the validation among 10 epochs on ResNet50 model, as we can see there is a strong positive correlation between training accuracy and testing accuracy among the 10 epochs, so we can conclude that the model overcomes the problem of overfitting during training and achieves a test accuracy, which is almost the same as the training accuracy.

The article "Human-Computer Interaction with Hand Gesture Recognition Using ResNet and MobileNet" was published in 2022. Journal: Comput Intell Neurosci.

We will also see other metrics to evaluate how our model individually performs with each class through the confusion matrix. As illustrated in Figure 17, the confusion matrix is a review of the projection outcomes on a classification task. The number of correct and inaccurate guesses is summarized by counting numbers and split down by class. The confusion matrix is made up of *N* ∗ *N* matrices, where *N* is the number of classes (32). Where the dark cells in the matrix correspond to low cell value and brighter cells correspond to high cell value, we can see in Figure 17 that the diagonal has the brighter cells (highest values), which means that most of the images are correctly predicted to its real class. It shows us that our model performs well for each class on the testing set.

### 5.1. Evaluation Metrics

Also, we used other different evaluation metrics as the precision and recall and F1-score in order to individually evaluate our model with respect to each class from the 32 Arabic alphabet sign classes as shown in Table 4.

Precision: It is also known as the positive predictive value. Accuracy is defined as the proportion of correct predictions divided by the total number of correct class values projected. Equation (14) is used to calculate the precision.
  (14) $$\begin{array}{c} \text{Precision}=\frac{\text{TruePositive}}{\text{TruePositive}+\text{FalsePositive}}. \end{array}$$
Recall: It is sometimes referred to as vulnerability. The recall is defined as the proportion of correct predictions divided by the number of correct class values. Equation (15) is used to calculate recall.
  (15) $$\begin{array}{c} \text{Recall}=\frac{\text{TruePositive}}{\text{TruePositive}+\text{FalseNegative}}. \end{array}$$
F1-score: The *F*-score or F-measure is another name for the F-score. The F1-score represents the balance between precision and recall. Only when the precision and recall numbers both are good, the F1-score grows high. F1-score values array from 0 to 1, and the greater the number, the greater the classification accuracy [10].

F1-score is calculated by (16)

(16) $$\begin{array}{c} \text{F}1-\text{score}=\frac{2*\text{Precision}*\text{Recall}}{\text{Precision}+\text{Recall}}. \end{array}$$

This table summarizes the results using the metrics we described in detail above, and we can see that the combined metric, which is F1-score, is high for all the 32 classes, which means that our model classifies all classes as very good on the test set.

Summary of our results with different models.

The highest accuracy was received when we ensembled the prediction of our trained models, and we achieved 98.2% accuracy on the test set as shown in Table 5.

The article "Human-Computer Interaction with Hand Gesture Recognition Using ResNet and MobileNet" was published in 2022. Journal: Comput Intell Neurosci.

### 5.2. Comparative Analysis

In order to help vocal people who do not know sign language and cannot communicate with deaf people and hearing-impaired people, which mainly communicate using sign language, a lot of research has been performed for developing systems to address this problem and facilitate the communication process with deaf and hearing-impaired people. There are many research studies performed all around the world from different countries and cultures as each culture has its own sign language, which differs from other cultures. In this review section, we will focus our analysis on research studies that target Arabic sign language.

We reviewed recent several studies that are highly related to our study. Some of these studies are shown in Table 6.

## 6. Discussion

In this study, sign language recognition is considered for detecting the Arabic alphabet. The purpose of this study is to assist hearing-impaired people by assisting them with modern technology. The dataset used in this study is ArASL2018, and it consisted of 54,000 images of 32 Arabic sign language alphabets. Various preprocessing techniques were applied to these images like reshaping, resizing, smoothing the images, and removing the noise. Apart from preprocessing, data augmentation techniques were also applied. These techniques would help in improving the model and the accuracy. Subsequently, preprocessing is performed. The images are resized to 64 ∗ 64 pixels and converted from grayscale images to three-channel images. We applied the median filter to the images, which acts as lowpass filtering in order to smooth the images and reduce noise, to make the model more robust when generalizing in real-life scenarios (images), and to avoid overfitting as possible. Different augmentation techniques are applied to the images. Then, the preprocessed image is fed into two different models, which are ResNet50 and MobileNetV2. ResNet50 and MobileNetV2 architectures were implemented together. We applied two different models to our experimentation, and these two models were pretrained on the Google ImageNet dataset. The first model ResNet50 achieved an accuracy on the test set of about 97.5%. The second model MobileNetV2 achieved an accuracy on the test set of about 97%. Finally, when we ensembled the predictions of these two models, and our accuracy increased to about 98.2%.

### 6.1. Samples of Real-Time Detection

In Figure 18 we can see the first 9 Arabic alphabets and their classification in real time, and we process the real-time video to predict the hand gesture in each frame and classify it to one of the alphabet classes.

The article "Human-Computer Interaction with Hand Gesture Recognition Using ResNet and MobileNet" was published in 2022. Journal: Comput Intell Neurosci.

### 6.2. Limitations in Real-Time Detection

Since all the dataset was taken in the same place and under the same lighting conditions and in the static background as discussed in the dataset section, in real time the model works best on bright or white background, and static or noncomplex backgrounds.

## 7. Conclusions

Hand movements have been an important part of communication since the beginning of time. Sign language, a visual form of communication, is based on hand movements. An insight study of convolutional neural network (CNN) design is specifically designed for hand motion sign language identification within that research. This technique is well described and provides greater classification results with less training sets than those of other current CNN models. In this investigation, VGG-11 and VGG-16 were also designed and evaluated to test the effectiveness of this system. A currently accessible American Sign Language (ASL) database is utilized to assess competence. The competence of the proposed system, VGG-11, and VGG-16 is experimentally evaluated in caparison to state structure techniques. Several effectiveness measures, in addition to accuracy, were used to assess the efficacy of the suggested task. The findings reveal that the proposed model outperforms previous techniques since it can classify a large number of signals with a low rate of error. The technique is also tested with the new data and shown to be the rotation and resizing robust. Here in this work, we trained a model, which will be able to classify the Arabic sign language, which consists of 32 Arabic alphabet sign classes. In images, sign language is detected through the pose of the hand. In this study, we proposed a framework that consists of two CNN models, and each of them is individually trained on the training set. The final predictions of the two models were ensembled to achieve higher results. Dataset: We worked on a dataset released in 2019 and called ArSL2018 launched at the Prince Mohammad Bin Fahd University, Al Khobar, Saudi Arabia, and we will talk about the details of this dataset in the next section. Summary of results: We achieved on the test set that we took from our whole data an accuracy of about 97% after applying many preprocessing techniques and different hyperparameters for each model, different augmentation techniques, etc.

## Figures and Tables

**Figure 1:** Representation of the Arabic sign language for Arabic alphabets.

**Figure 2:** Distribution of ArSL2018 dataset classes.

**Figure 3:** Augmentation through horizontal flipping.

**Figure 4:** Augmentation through rotating images.

The article "Human-Computer Interaction with Hand Gesture Recognition Using ResNet and MobileNet" was published in 2022. Journal: Comput Intell Neurosci.

**Figure 5:** Augmentation through shearing images.

**Figure 6:** Augmentation through changing images.

**Figure 7:** Without skip connection.

**Figure 8:** Skip connection.

**Figure 9:** ResNet50 residual block [31].

**Figure 10:** MobileNetV2 building block [32].

**Figure 11:** Standard convolution [33].

**Figure 12:** Depthwise convolution [34].

**Figure 13:** Pointwise convolution [35].

**Figure 14:** Alphabet recognition flowchart.

**Figure 15:** Model accuracy.

**Figure 16:** Model loss.

**Figure 17:** Confusion matrix.

**Figure 18:** Real-time Arabic sign alphabet recognition.

**Table 1:** Dataset classes and their labels and number of images.

#	Letter name in English script	Letter name in Arabic script	# of images
1	Alif	(ألف) أ	1672
2	Ba	(باء) ب	1791
3	Ta	(تاء) ت	1838
4	Tha	(ثاء) ث	1766
5	Jim	(جيم) ج	1552
6	Ha	(حاء) ح	1526
7	Kha	(خاء) خ	1607
8	Dal	(دال) د	1634
9	Dhal	(ذال) ذ	1582
10	Ra	(راء) ر	1659
11	Zay	(زين) ز	1374
12	Sin	(سين) س	1638
13	Shin	(شين) ش	1507
14	Sad	(صاد) ص	1895
15	Dad	(ضاد) ض	1670
16	Ta	(طاء) ط	1816
17	Za	(ظاء) ظ	1723
18	Ayn	(عين) ع	2114
19	Ghayn	(غين) غ	1977
20	Fa	(فاء) ف	1955
21	Qaf	(قاف) ق	1705
22	Kaf	(كاف) ك	1774
23	Lam	(لام) ل	1832
24	Mim	(ميم) م	1765
25	Nun	(نون) ن	1819
26	Ha	(هاء) هـ	1592
27	Waw	(واو) و	1371
28	Ya	(يا) ى	1722
29	Taa	(ة) ة	1791
30	Ai	(ال) ال	1343
31	Laa	(لا) لا	1746
32	Yaa	(ياء) ي	1293

**Table 2:** Summary of the modified ResNet50 model.

Transfer learning	Pretrained on Google ImageNet dataset
Number of layers	50 layer of ResNet50 architecture +3 sequential layers (2 fully connected layers + 1 softmax layer). Therefore, the total number of layers is 53 layers
Number of neurons in fully connected layers	1,024 neurons in the 1 fully connected layer, 512 neurons in the 2nd fully connected layer, and 32 neurons in the last layer (softmax layer)
Activation function	ReLu activation function
Optimizer	Adam optimizer with 0.0001 learning rate
Dropout	Dropout value used for the fully connected layers is 0.5
Batch size	32
Loss function	Categorical loss entropy
Number of epochs	10 epoch
Total no. of parameters	Total params: 32,495,648- trainable params: 32,450,208- nontrainable params: 45,440

**Table 3:** Summary of the modified MobileNetV2 model.

Transfer learning	Pretrained on Google ImageNet dataset.
Number of layers	53 layers0 of MobileNetV2 architecture +3 sequential layers (2 fully connected layers + 1 softmax layer).Therefore, the total number of layers is 56 layers
Number of neurons in fully connected layers	1,024 neurons in the 1st fully connected layer, 512 neurons in the 2nd fully connected layer, and 32 neurons in the last layer (softmax layer)
Activation function	ReLu activation function
Optimizer	Adam optimizer with 0.0005 learning rate
Dropout	Dropout value used for the fully connected layers is 0.5
Batch size	32
Loss function	Categorical loss entropy
Number of epochs	15 epoch
Total no. of parameters	Total params: 8,043,104- trainable params: 8,008,992- nontrainable params: 34,112

The article "Human-Computer Interaction with Hand Gesture Recognition Using ResNet and MobileNet" was published in 2022. Journal: Comput Intell Neurosci.

**Table 4:** Model evaluation metrices.

Alphabets	Precision	Recall	F1-score
Ain	0.97	0.99	0.98
Al	1	0.97	0.98
Aleff	0.85	1	0.92
Bb	0.93	0.98	0.95
Dal	0.84	0.99	0.91
Dha	0.94	0.95	0.94
Dhad	0.97	0.98	0.98
Fa	0.97	0.9	0.94
Gaaf	0.95	0.95	0.95
Ghain	0.99	0.99	0.99
Ha	0.91	0.97	0.94
Haa	0.96	0.97	0.97
Jeem	0.95	1	0.97
Kaaf	0.97	0.98	0.98
Khaa	0.99	0.96	0.97
La	0.99	0.98	0.99
Laam	1	1	1
Meem	0.97	0.98	0.98
Nun	1	0.95	0.97
Ra	0.94	0.89	0.91
Saad	0.99	0.92	0.95
Seen	0.99	0.97	0.98
Sheen	0.97	0.99	0.98
Ta	0.98	0.88	0.93
Taa	0.94	0.93	0.93
Thaa	0.95	0.93	0.94
Thal	0.97	0.91	0.94
Toot	0.99	1	1
Waw	0.99	0.95	0.97
Ya	0.99	1	1
Yaa	0.99	0.99	0.99
Zay	0.98	0.92	0.95

**Table 5:** Final results.

Method	Testing accuracy (%)
ResNet50	97.5
MobileNetV2	97.1
ResNet50 + MobileNetV2	98.2

**Table 6:** Comparison of related work.

Reference	Feature extraction	Classification	Accuracy (%)	Number of classes
[28]	(i) CNN Model		90	31 class
[36]	(ii) CNN Model		88.87	28 class
[29]	(i) Hand shape-based description, where each hand image was described by a vector consisting of 15 values where the values represent the key points locations	(i) KNN classifier-Naïve-Bayesian	97.548	28 class
Our research study	(i) ResNet50 and MobileNetV2		98.2	32 class

## Data Availability

The data that support the findings of this study are available in paper “Latif, Ghazanfar; Alghazo, Jaafar; Mohammad, Nazeeruddin; AlKhalaf, Roaa; AlKhalaf, Rawan (2018),” “Arabic Alphabets Sign Language Dataset (ArASL),” Mendeley Data, V1, doi: 10.17632/y7pckrw6z2.1.
